# Cytocompatibility and biocompatibility of nanostructured carbonated hydroxyapatite spheres for bone repair

**DOI:** 10.1590/1678-775720150122

**Published:** 2015

**Authors:** Mônica Diuana CALASANS-MAIA, Bruno Raposo de MELO, Adriana Terezinha Neves Novellino ALVES, Rodrigo Figueiredo de Brito RESENDE, Rafael Seabra LOURO, Suelen Cristina SARTORETTO, José Mauro GRANJEIRO, Gutemberg Gomes ALVES

**Affiliations:** 1 - Universidade Federal Fluminense, Faculdade de Odontologia, Departamento de Cirurgia Oral, Núcleo de Pesquisa Clínica em Odontologia, Niteroi, RJ, Brazil.; 2 - Universidade Federal Fluminense, Faculdade de Odontologia, Niteroi, RJ, Brazil.; 3 - Instituto Nacional de Metrologia, Qualidade e Tecnologia, Programa de Bioengenharia, Duque de Caxias, Rio de Janeiro, Brazil,; Universidade Federal Fluminense, Faculdade de Odontologia, Niteroi, RJ, Brazil.; 4 - Universidade Federal Fluminense, Instituto de Biologia, Departamento de Biologia Celular e Molecular, Niteroi, RJ, Brazil

**Keywords:** Hydroxyapatite, Bone repair, Biocompatibility testing, RANKL/OPG, Rats

## Abstract

**Objective:**

The aim of this study was to investigate the *in vitro* and *in vivo* biological responses to nanostructured carbonated hydroxyapatite/calcium alginate (CHA) microspheres used for alveolar bone repair, compared to sintered hydroxyapatite (HA).

**Material and Methods:**

The maxillary central incisors of 45 Wistar rats were extracted, and the dental sockets were filled with HA, CHA, and blood clot (control group) (n=5/period/group). After 7, 21 and 42 days, the samples of bone with the biomaterials were obtained for histological and histomorphometric analysis, and the plasma levels of RANKL and OPG were determined via immunoassay. Statistical analysis was performed by Two-Way ANOVA with *post-hoc* Tukey test at 95% level of significance.

**Results:**

The CHA and HA microspheres were cytocompatible with both human and murine cells on an *in vitro *assay. Histological analysis showed the time-dependent increase of newly formed bone in control group characterized by an intense osteoblast activity. In HA and CHA groups, the presence of a slight granulation reaction around the spheres was observed after seven days, which was reduced by the 42^nd^ day. A considerable amount of newly formed bone was observed surrounding the CHA spheres and the biomaterials particles at 42-day time point compared with HA. Histomorphometric analysis showed a significant increase of newly formed bone in CHA group compared with HA after 21 and 42 days from surgery, moreover, CHA showed almost 2-fold greater biosorption than HA at 42 days (two-way ANOVA, p<0.05) indicating greater biosorption. An increase in the RANKL/OPG ratio was observed in the CHA group on the 7^th^ day.

**Conclusion:**

CHA spheres were osteoconductive and presented earlier biosorption, inducing early increases in the levels of proteins involved in resorption.

## INTRODUCTION

The application of procedures for bone regeneration is becoming a daily practice in orthopedic and maxillofacial surgery, motivated by the wide acceptance of dental implants as an option for oral rehabilitation. For instance, dento-alveolar trauma usually demands reconstruction of the alveolar crest before an implant can be put in place^13^. Several studies have demonstrated the potential for the use of autogenous bone grafts for bone regeneration due to the bone-forming cells potentially harbored in such grafts and their ability to release substances that induce bone formation (osteogenesis) as well as to serve as a scaffold for bone formation (osteoconductivity)^11^ ^,^ ^26^. However, difficulties in obtaining autogenous bone grafts and limitations, such as postoperative discomfort in patients, donor site morbidity, and the limited availability of graft materials, as well as ethical issues and the possibility of disease transmission from allogeneic or xenogeneic grafts, have motivated researchers to develop synthetic or alloplastic materials^1^ ^,^ ^16^ ^,^ ^17^ ^,^ ^22^. In this context, calcium phosphates present interesting features related to bone-targeting applications such as excellent bioactivity, the ability to bond directly to bone, and osteoconductivity. In addition, calcium phosphates can be resorbed, showing solubility rates that are dependent on their composition and microstructural features^10^.

Hydroxyapatite (HA), Ca_10_(PO_4_)_6_(OH)_2_, is the main mineral component of bone and teeth, and has been widely applied as a biomaterial due to its well-known bioactivity and osteoconductivity, even though HA ceramics are poorly degradable under physiological conditions^12^. Nevertheless, its structure allows isomorphic cationic and anionic substitutions to be easily introduced^20^, which can alter the crystallinity, morphology, lattice parameters, crystal size, stability, bioactivity, biocompatibility, and osteoconductivity of HA^4^, offering alternatives for the development of improved materials. For instance, changes in the chemical composition of HA induced through partial substitution of the phosphate group (PO_4_) with a carbonate group (CO_3_) lead to the formation of a B type carbonated hydroxyapatite (CHA). CHA has been proposed as an alternative material for bone regeneration not only due to its similarity to the mineral phase of calcified tissue, but mainly because this material may overcome limitations related to crystallinity and low solubility, and therefore extend the therapeutic capacity of HA^12^ ^,^ ^28^. Moreover, the alginate was included in the material, since it is a biocompatible and soluble biopolymer, commonly used to allow the formation of hydroxyapatite microspheres; it also modulates the degradation rate of the biomaterial^28^.

With the progress of nanotechnology, another important development in materials science has been the synthesis of HA-based ceramics at the nanometric level, producing HA nanoparticles, blocks, coatings, and nanostructured materials^2^. The rationale for the use of nanostructured CHA (produced from particles smaller than 100 nm) is based on the fact that natural bone formation involves particles of a similar nanometric size^18^ ^,^ ^27^. Nanoparticles are also expected to exhibit improved bioactive properties^28^. Recent studies have shown that nanostructured calcium phosphates display better selective protein adsorption ability *in vivo*, and can also regulate the cascade of expression of specific intracellular genes and cell behaviors, thus inducing the regeneration of specific tissues^23^. These materials can be synthesized through diverse methodologies, including the precipitation of nanometric particles at relatively low processing temperatures (below 10°C) via a procedure that may even produce nanostructured carbonated hydroxyapatite^28^. However, there are few evidences regarding the bioactivity of low crystalline nanostructured carbonated hydroxyapatite and the impact on the outcome of alveolar bone repair during oral rehabilitation procedures. Therefore, the aim of the present study was to evaluate the biocompatibility of spheres of nanostructured carbonated hydroxyapatite/calcium alginate, employing stoichiometric sintered hydroxyapatite spheres as a reference and comparing their effectiveness in alveolar bone repair, while determining their correlation with two relevant plasma biochemical markers of the bone remodeling/resorption process, namely RANKL (Receptor Activating Factor Nuclear Kappa-β) and OPG (Osteoprotegerin).

## MATERIAL AND METHODS

### Material

Carbonated hydroxyapatite powder was synthesized from aqueous solutions of extra-pure calcium nitrate tetra-hydrate, dihydrogen ammonium phosphate, and ammonium carbonate (Merck, Taquara, Rio de Janeiro, Brazil). The reagents were mixed and maintained at 5°C for 2 h at pH=13 in the presence of KOH with a stoichiometry of 1.6<Ca/P<2.0. The X-ray diffraction pattern of the CHA powder (Figure 1) presented broad peaks due to the nanostructured and poorly crystalline nanostructure compared with HA. The carbonated hydroxyapatite and hydroxyapatite powders (<74 µm) were mixed in a sodium alginate solution (Sigma Aldrich^®^/Fluka Biochemika^®^, St. Louis, Missouri, USA), 1% wt with light agitation of calcium chloride (CaCl_2_, 0.15 M) at room temperature (approximately 20°C) to obtain microspheres with different diameters as a result of the ionic interchange between the sodium alginate and calcium chloride; it also modulates the degradation rates of the biomaterial. The microspheres were removed from the solution, sieved (425< 425<Ø<550 μm), washed in MilliQ water (MilliQ^®^, Millipore Corporation, Billerica, Massachusetts, USA) and dried in an oven at 70°C for 24 h (Figure 2). The HA samples were sintered at 1000°C for 27 hours to obtain a crystalline biomaterial, and the CHA spheres were not thermally treated. The samples were synthesized and characterized at the Brazilian Center of Physics Research. The materials were sterilized by gamma radiation (25 kGrays), according to ISO 11137 (Sterilization of health care-products-Radiation) at the Nuclear Instrumentation Laboratory, COPPE, Rio de Janeiro Federal University (the biomaterial synthesis is under patent process).

**Figure 1:** X-Ray Diffraction pattern (XRD) of the carbonated hydroxyapatite (CHA) powder. Observe broad peaks due to the nanostructured and poorly crystalline character of the CHA

**Figure 2:** Scanning Electron Microscopy (SEM) micrographs. A: Carbonated hydroxyapatite (CHA) spheres; B: CHA spheres surface, both without thermal treatment; C: Hydroxyapatite (HA) spheres, and D: HA spheres surface. A and C: 100X magnification, and B and D: 1,000X magnification. Scale bars of 1mm (A and C) and 100 µm (B and D)

### *In vitro* analysis – multiparametric cytotoxicity assay

Prior to animal testing, the cytocompatibility of the materials employed in this study was evaluated in accordance with the recommendations contained in ISO 7405:2008 regarding the assessment of dental materials. Extracts were prepared via the immersion of 200 mg of biomaterial spheres in 10 mL of culture medium (DMEM, Dulbelcco, St. Louis, Missouri, USA) by 24 hours at 37°C. Subsequently, these extracts were added to subcultures of either (i) a murine pre-osteoblast cell line (MC3T3-E1) or (ii) primary human osteoblasts (Hob) obtained from the collection at Clinical Research Unit-Antonio Pedro University Hospital. The cells were seeded into 96-well culture plates at a density of 10^4^ cells/well, and incubated in the presence of the extracts for 24 hours at 37°C under 5% CO_2_. At the end of incubation period, the cells were washed with PBS, and viability tests were performed.

Cell viability was assessed using a multiparametric method^8^ that allows various parameters related to survival to be analyzed in the same exposed cells. These parameters included mitochondrial activity (XTT Test), membrane integrity (Neutral Red Uptake Assay, NR) and cell densities (Crystal Violet Dye Exclusion assay, CVDE). For these tests, commercial kits were used (In Cytotox, Xenometrix, Allschwil, Arlesheim, Switzerland).

### *In vivo* analysis of biocompatibility

#### Experimental groups

All procedures were carried out in accordance with conventional guidelines in the Guide for the Care and Use of Laboratory Animals (US National Institutes of Health 85-23, revised 1996). The local Institutional Animal Care and Use Committee of Fluminense Federal University, Niteroi, Brazil (protocol number 194/10) approved all experimental protocols.

Three-month-old male Wistar rats weighing approximately 250 g were maintained under standard conditions with free access to food and water. A total of 45 animals were divided into 3 groups and examined after different experimental periods (7, 21 or 42 days after surgery). Fifteen animals were distributed into three experimental groups, with 5 of the rats surgically treated with CHA (CHA group), 5 treated with the reference material (HA group), and 5 to control group (non-grafted alveolar sockets).

#### Surgical procedures

All animals were anesthetized with ketamine (20 mg/kg) (Virbac, Jurubatuba, SP, Brazil) and xylazine (1 mg/Kg) (FortDodge, São Cristovão, RJ, Brazil). Subsequently, syndesmotomy of periodontal tissue was performed using a syndesmotome (Duflex^®^, Rio de Janeiro, Rio de Janeiro, Brazil), and the upper-right incisor was extracted with a clinical probe adapted to this tooth (Figure 3A). The dental sockets were filled with nanostructured hydroxyapatite carbonated (CHA group), hydroxyapatite (HA group), or blood clot (control group), and sutured with Vicryl 4-0 (Johnson & Johnson Medical Ltd., Blue Ash, Ohio, United States) (Figure 3B). The rats were anesthetized and killed with the same anesthetic agents used for surgical implantation at the end of the experimental period, either 7, 21 or 42 days after surgery, and samples containing the biomaterials were removed.

**Figure 3:** Surgical procedures for biomaterials implantation: A: The maxillary right incisor was extracted, and B: The socket was filled with spheres of biomaterials according to the experimental group.

#### Descriptive histological analysis

Noncalcified samples were histologically processed via embedding in paraffin, cut into 5 μm-thick sections and stained with Hematoxylin and Eosin (HE) for light microscopy assessment (Olympus BX43, Tokyo, Kanto, Japan). The reaction of the cells to the biomaterials was observed, focusing on the intensity and nature of the inflammatory response and the presence of necrosis, fibrous connective tissue and neoformed bone in direct contact with the graft.

#### Histomorphometric analysis

For histomorphometric analysis, a light microscope (Olympus BX43, Tokyo, Kanto, Japan) with 10x of magnification was used. The microscope was connected to a computer and each HE-stained histological slice corresponding to the alveolar region was captured by scanning by Image acquisition software (Cellsens^®^ 1.9 Digital, Tokyo, Kanto, Japan). One expert observer analysed ten non-consecutive images of each section. With the Image-Pro Plus^®^ 6.0 (Media Cybernetics, Silver Spring, Maryland, USA), a grid of 200 points were superimposed on captured field, permitting the determination of newly formed bone and the residual biomaterial. The bone volume density (BV/TV%) was calculated by bone volume over total volume, indicating the fraction of volume of interest that was occupied by bone. For biomaterial volume density (BiomatV/TV%), the same calculation method was applied. The areas were expressed in percentage.

#### Determination of plasma RANKL and OPG levels

Blood samples (5 mL) were collected from each animal via cardiac puncture following intraperitoneal anesthesia with ketamine (75 mg/kg) and xylazine (5 mg/kg). The samples were subsequently centrifuged at 1,700 rpm for 10 min, without hemolysis, and the plasma was collected and stored in a freezer at -80°C for posterior analysis. The total plasma levels of RANKL and OPG were assessed in immunoassays based on xMAP technology with a Luminex S200 Multiplex Flow Luminometer (Luminexcorp, Austin, Texas, USA), employing commercial kits (Rat Bone Panel 1 Milliplex MAP kit, Millipore, Billerica, Massachusetts, USA). The results were analyzed using Xponent v. 3.0 software (Luminexcorp, Austin, Texas USA).

## Statistical analysis

The mean values and standard deviations obtained in each cytotoxicity assay (n=3 trials in quintuplicate) were tested for normality according to D’Agostino and Pearson’s omnibus. Upon verification of a normal distribution, two-way ANOVA was conducted together with Tukey’s *post-hoc* test. The significance level was set at p=0.05. Also, after the normality test, a quantitative description with means and confidence interval (CI) of BV/TV% and BiomatV/TV% was performed. The analysis of variance of two-way ANOVA and Tukey’s *post-hoc* test was applied, and two assignable sources of variation - groups and periods - were evaluated. The significance level was set at p=0.05. Both *in vitro* and *in vivo* analyzes were performed using Prism Graph Pad 6.3 software (Inc. La Jolla, California, USA).

## RESULTS

### *In vitro* evaluation of biocompatibility

The cytotoxicity assays, performed using murine pre-osteoblasts (MC3T3-E1), showed that both the CHA and HA groups were cytocompatible, with more than 75% cell survival observed when compared to the experimental control group (cells exposed to culture medium), as recommended by international standards (ISO 7405:2008). Moreover, the results observed in the CHA group were similar to those of the experimental and negative control (polystyrene) groups for the evaluated parameters. These findings were obtained in both murine (Figure 4) and human primary bone cells (Figure 5). It could also be observed that both the positive and negative controls behaved as expected, with polystyrene being highly cytocompatible, while latex extracts dramatically reduced cell viability in all assays. Therefore, the materials were considered to be suitable for subsequent *in vivo* tests*.*

**Figure 4:** Multiparametric cytotoxicity assay with murine MC3T3-E1 cells. Results showed as percentage of control group (Control; exposure to DMEM). * ≠ all the other groups (p<0.05)

**Figure 5:** Multiparametric cytotoxicity assay with human osteoblastic cells. Results showed as percentage of control group (Control; exposure to DMEM). * ≠ all the other groups (p<0.05)

### Histological analyses

Morphological analysis was performed at light microscope after hematoxylin-eosin staining. The Figures 6, 7 and 8 contain representative photomicrographs of alveolar socket from each implanted biomaterials and control group at magnification of 4 and 40X.

**Figure 6:** Representative photomicrographs of alveolar socket after 7 days. A and B: Control group; C and D: HA group; E and F: CHA group. The small squares identified by B, D and F are displayed at 40-fold magnification adjacent to the figures with lower magnification (Figures A, C and E, respectively). Pre-existing bone (PEB); Connective tissue (CT); Osteoblasts pavement (black arrow); serum hemorrhagic exudate (*); Newly formed bone (NFB); Neutrophilic infiltrate (n); Osteoid (o); hydroxyapatite (HA); nanostructured carbonated hydroxyapatite/calcium alginate (CHA). Hematoxylin and eosin stained.

In seven days, the control group showed few trabeculae of newly formed bone with osteoblasts pavement on periphery, interspersed by connective tissue containing serum hemorrhagic exudate (Figures 6A and 6B). Both biomaterial groups presented the dental socket filled by biomaterial spheres (Figures 6C and 6E) permeated by connective tissue characterized by granulation reaction. In HA group, focal areas of scanty neutrophilic infiltrate surrounding the spheres were observed (Figure 6D). In CHA group, an initial osteoid deposition surrounding the spheres was found (Figure 6F).

At 21-day time point, the control group presented more trabeculae of newly formed bone than 7-day time point, interspersed by connective tissue and hemorrhagic exudate. The newly formed bone was surrounded by osteoblasts line (Figures 7A and 7B). The spheres of HA group were not dispersed (Figure 7C) as in the first period yet. In the CHA group, the same spheres presented a smaller diameter than at day 7 (Figure 7E), and displayed some areas of biomaterial particles suggesting a biosorption. Islands of newly formed bone surrounding the biomaterials spheres were observed at high magnification at both groups (Figures 7D and 7F).

**Figure 7:** Representative photomicrographs of alveolar socket after 21 days. A and B: Control group; C and D: HA group; E and F: CHA group. The small squares identified by B, D and F are displayed at 40-fold magnification adjacent to the figures with lower magnification (Figures A, C and E, respectively). Pre-existing bone (PEB); Connective tissue (CT); Osteoblasts pavement (black arrow); hemorrhagic exudate (*); Newly formed bone (NFB); hydroxyapatite (HA); nanostructured carbonated hydroxyapatite/calcium alginate (CHA). Hematoxylin and eosin stained

After 42 days, the alveolar socket of control group was almost filled by newly formed bone interspersed by connective tissue and remnant hemorrhagic exudate (Figures 8A). At high magnification, there was observed the trabeculae periphery surrounded by a large osteoblasts pavement (Figures 8B). Both groups of biomaterials presented a reduction of biomaterial amount compared with previous periods (Figures 8C and 8E). The HA group showed regions of newly formed bone surrounding the spheres (Figures 8D). A reduction of the amount of discernible CHA spheres could be observed between 7 and 42 days (Figures 6E and 8E). A considerable amount of newly formed bone was observed surrounding the spheres and the biomaterials particles (Figures 8F). Moreover, the final amount of CHA, observed after 42 days, was smaller compared to the amount of HA at the same experimental time (Figures 8C and 8E), and in CHA group the newly formed bone seems to be in higher amount than in HA group (Figures 8D and 8F).

**Figure 8:** Representative photomicrographs of alveolar socket after 42 days. A and B: Control group; C and D: HA group; E and F: CHA group. The small squares identified by B, D and F are displayed at 40-fold magnification adjacent to the figures with lower magnification (Figures A, C and E, respectively). Pre-existing bone (PEB); Connective tissue (CT); Osteoblasts pavement (black arrow); hemorrhagic exudate (*); Newly formed bone (NFB); hydroxyapatite (HA); nanostructured carbonated hydroxyapatite/calcium alginate (CHA). Hematoxylin and eosin stained

### Histomorphometric analysis

#### BV/TV% (p<0.05)

Histomorphometric analysis showed a significant increase of BV/TV% in CHA group compared with HA after 21 and 42 days from surgery. Moreover, we found a time dependent increase of BV/TV% in CHA group at 42 and 21 days compared with 7-day time point and 42 days compared with 21-day time point. The HA showed a significant increase at 21-day and 42-day compared with 7-day time point, following by a stabilization of bone formation at 42 days compared with 21 days. The control group presented a significant increase of BV/TV% compared with HA in all experimental groups, however, compared with CHA group, the difference was observed only at 42 days (p<0.05) (Figure 9A).

**Figure 9:** The bone volume density (BV/TV%) (A), and biomaterials volume density (BiomatV/TV%) (B) after 7, 21, and 42 days of implantation. (a) significant statistical differences between hydroxyapatite (HA) or nanostructured carbonated hydroxyapatite/calcium alginate (CHA) compared with control group at the same experimental period; (b) significant statistical differences between CHA and HA at the same experimental period; (*) significant statistical difference between the same group at different experimental periods (two-way ANOVA, p<0.05). Results are shown as mean percentages±confidence interval

#### BiomatV/TV%

The Figure 9B presents a time-dependent trend of reduction in BiomatV/TV% presence in both groups after biomaterials implant. A significant decrease in BiomatV/TV% of CHA at 42 days after surgery compared with 7 and 21 days was found, while HA showed a reduction in biomaterial at 42 days compared with only 7 days. Also, CHA group presented a higher biosorption of BiomatV/TV% compared with HA at 42 days. Specifically, CHA showed almost 2-fold greater biosorption than HA at 42 days (p<0.05).

#### RANKL/OPG analysis

OPG levels significantly decreased between 7 and 42 days in the HA group (p<0.05), whereas no significant effect of time was found for this molecule in the CHA group. The RANKL concentration was significantly higher (p<0.05) in the CHA group compared to the HA group after 7 days, and decreased from 7 to 42 days, whereas it remained stable at lower levels for the HA group. The RANKL/OPG ratio was higher in the CHA group compared to the HA group after 7 days, but not after 42 days. There was no significant difference in this ratio between 7 and 42 days in the CHA group (Figure 10).

**Figure 10:** Serum concentrations assay of RANKL/OPG in operated rats after 7 and 42 days. Abbreviations: CHA=carbonated hydroxyapatite/sodium alginate; HA=stoichiometry hydroxyapatite. Bar ≠ between groups (p<0.05); * ≠ all the other groups (p<0.05)

## DISCUSSION

The use of spheres or granules to biocompatible materials for clinical use has been previously proposed^6^ ^,^ ^21^ ^,^ ^24^, as they may be injectable and moldable, and simulate a porous environment for increased osteoconductivity. In this context, carbonated nanostructured hydroxyapatite/sodium alginate spheres may be a promising biomaterial for bone replacement. Carbonated hydroxyapatite is described as more bioactive and soluble than stoichiometric HA, mainly due to properties such as its particle size, surface area, and morphology. Also, nanostructured CHA with low crystallinity may present improved characteristics that are desirable in many fields, including tissue engineering and dental implantology^28^. This report presents an *in vitro* and *in vivo* analysis of the biocompatibility of nanostructured carbonated hydroxyapatite/sodium alginate as a bone substitute in the alveolar bones of rats.

One of the methodological advantages of the *in vitro* model applied in the present work was that, within the same group of treated cells, three different parameters were evaluated. The relevance of this difference becomes evident when we consider that the results obtained using only one method are often overestimated or underestimated due to interference or methodological limitations. Previous studies have revealed conflicts between the results obtained with tetrazolium-based assays and other parameters^3^ ^,^ ^9^. Therefore, while the XTT assay showed that neither of the tested materials affects cell metabolism, the other assays ensured that membrane integrity (NR) and proliferation (CVDE assay) were also preserved upon exposure to HA and CHA. In fact, there is not a general consensus on nanoparticle toxicity (as it is totally dependent of the physicochemical nature of the material). For instance, literature indicates that the toxicity of nanoHA is closely related to particle size^8^. The spheres of the present work are nanostructured (i.e., synthesized from nanocrystals, even though the final product is on the micrometric scale). Therefore, there was no direct expectancy of cytotoxicity. Nevertheless, in order to guarantee the absence of significant adverse effects, three different cell viability parameters were successfully accessed *in vitro*, prior to animal testing.

Another important feature of *in vitro* analyses is the choice of the cell type to be exposed to the tested material. MC3T3-E1 cells are pre-osteoblasts that are able to produce a mineral matrix when subjected to the correct stimulus. Because these cells are of murine origin, the *in vitro* test was able to reduce the risk of exposure of the rats during the *in vivo* steps of the present work. However, our model also included human osteoblasts in primary culture. These cells exhibit a greater proximity to the end-use of the materials because the integrity of their genome is often preserved (in contrast to transformed or tumoral cell lines), and osteoblasts are among the cell types that are intended to interact with the material during new bone formation^20^.

Our *in vivo *results showed that nanostructured CHA and stoichiometric HA grafts are biocompatible with bone repair in rats. It was observed through histological analysis that CHA group showed intense bone formation in 42 days, displaying layers of identifiable osteoblastic cells and large. Moderate inflammatory infiltrate was observed in both biomaterials groups, especially seven days after surgery, although they decreased by the 42^nd^ day, indicating the absence of an undesirable chronic inflammatory response. The amount of identifiable biomaterial also decreased from 7 to 42 days, mainly in the CHA group, indicating greater absorption of the material, probably due to a high concentration of phagocytic cells around the biomaterial. The greater absorption of CHA observed during this study corroborates previous studies, showing that CHA exhibits higher solubility and absorption due to its lower crystallinity^14^ ^,^ ^15^. In fact, nanostructured CHA spheres present greater *in vivo* resorption, even when grafted in maxillary sinus^28^. Analysis of histological slides stained with HE showed that CHA is also osteoconductive, leading to centripetal bone formation (towards the center of the defect).

Several proteins may be explored as markers of the bone remodeling process, e.g.: bone sialoprotein (BSP), osteoclast-specific enzymes, such as tartrate-resistant acid phosphatase or cathepsin K, type I collagen, osteocalcin, alkaline phosphatase, and others. Among those, the ratio of the important bone regulatory proteins RANKL and OPG represent an important tool for the understanding of the osteoclast-mediated resorption process of both bone and biomaterials. The RANKL/OPG system is described as a dominant mediator of osteoclastogenesis^25^. A better understanding of this system led to a new perspective regarding the molecular biology of osteoclasts and bone homeostasis. Specifically, the interaction between the osteoblast-secreted protein RANKL and the osteoclast receptor RANK is required for osteoclast differentiation and proliferation, while OPG acts as a soluble receptor and an antagonist to RANKL, preventing its binding to and activation of RANK^19^. The results of the present study showed that grafting with CHA induced an increase in RANKL production within one week, shifting the RANKL/OPG balance to favor resorption. These findings suggested that resorption of this biomaterial occurred in the early days following grafting, which was not observed in the HA group. This process could be involved in reducing the amount of the biomaterial present because osteoclasts release acid (H^+^), as well as other agents that dissolve crystals of calcium salts^26^, and may act to solubilize calcium phosphate from the biomaterial, favoring its absorption. Other *in vivo* and *in vitro* studies have shown that CHA (despite not being nanostructured) is preferentially resorbed by osteoclasts^14^ ^,^ ^15^. However, even though there was an increase in the number of multinucleated cells observed around the biomaterial, other tests must be performed to verify their identity as osteoclasts. It is important to note that other studies^30^ have demonstrated an increase in the RANK/OPG ratio in rats exposed to more-absorbable calcium phosphates, through a process that remains to be elucidated but seems to be associated with the levels of parathyroid hormone. Nevertheless, the present results may provide further evidence of increased biosorption of nanostructured CHA compared to stoichiometric crystalline HA.

## CONCLUSION

Based on these results we can conclude that spheres of nanostructured CHA are cytocompatible with both murine and human primary bone cells. This material presented biocompatibility and improved osteoconductive and biosorption properties when compared with stoichiometric hydroxyapatite regarding the alveolar bone repair in dental sockets. The increased resorption and the initial release of molecules involved in the activation of bone remodeling may indicate desirable properties of biomaterials, intended for their use in bone therapy and bone replacement following dental trauma prior to implantation surgery.
